# Deep Transfer Learning-Based Foot No-Ball Detection in Live Cricket Match

**DOI:** 10.1155/2023/2398121

**Published:** 2023-06-20

**Authors:** Sudhakar Das, Tanjim Mahmud, Dilshad Islam, Manoara Begum, Anik Barua, Mohammad Tarek Aziz, Eshatur Nur Showan, Lily Dey, Eipshita Chakma

**Affiliations:** ^1^Rangamati Science and Technology University, Rangamati, Bangladesh; ^2^Chattogram Veterinary and Animal Sciences University, Chittagong, Bangladesh; ^3^Port City International University, Chittagong, Bangladesh; ^4^International Islamic University Chittagong, Chittagong, Bangladesh; ^5^University of Chittagong, Chittagong, Bangladesh

## Abstract

Automation in every part of life has become a frequent situation because of the rapid advancement of technology, mostly driven by AI technology, and has helped facilitate improved decision-making. Machine learning and the deep learning subset of AI provide machines with the capacity to make judgments on their own through a continuous learning process from vast amounts of data. To decrease human mistakes while making critical choices and to improve knowledge of the game, AI-based technologies are now being implemented in numerous sports, including cricket, football, basketball, and others. Out of the most globally popular games in the world, cricket has a stronghold on the hearts of its fans. A broad range of technologies are being discovered and employed in cricket by the grace of AI to make fair choices as a method of helping on-field umpires because cricket is an unpredictable game, anything may happen in an instant, and a bad judgment can dramatically shift the game. Hence, a smart system can end the controversy caused just because of this error and create a healthy playing environment. Regarding this problem, our proposed framework successfully provides an automatic no-ball detection with 0.98 accuracy which incorporates data collection, processing, augmentation, enhancement, modeling, and evaluation. This study starts with collecting data and later keeps only the main portion of bowlers' end by cropping it. Then, image enhancement technique are implied to make the image data more clear and noise free. After applying the image processing technique, we finally trained and tested the optimized CNN. Furthermore, we have increased the accuracy by using several modified pretrained model. Here, in this study, VGG16 and VGG19 achieved 0.98 accuracy and we considered VGG16 as the proposed model as it outperformed considering recall value.

## 1. Introduction

Cricket is the second-most well-liked sport [1], with 2.5 billion spectators, just behind soccer/football, which has 3.5 billion fans [2]. Two teams of eleven players each compete in cricket, and each team is focused on winning. Two umpires are assigned to each end of the field to oversee the match (the end for bowlers and the end for strikers). The umpire must guarantee that the game is played in line with the laws [3]. The umpire's choice affects crucial rules. In a game, anything can happen in a split second, and a poor choice might significantly change the outcome. If a bad decision has an impact on the game, it has an impact on the entire fan base. Several regulations exist to make the game of cricket fair to both batters and bowlers, one of which is the no ball rule. No-ball rulings are the most difficult to forecast of all umpire judgments. Unlawful deliveries to a batter are known as “no balls” in cricket. There are many forms of no balls in cricket including front foot no ball, touching the return crease, a full toss no ball, uninformed change in bowling style, throwing the ball before delivery, chucking, fielding related no balls, wicket-keeping-related no ball, if the bowlers touch the wickets, and if the ball does not reach the batter [4]. This choice could result in a victory for one team or a defeat for the opposing team. A no-ball throw results in the addition of one run, or two under some rules, to the batting team's total score, and an additional ball must be bowled [5]. Therefore, it is vital to choose prudently in a no-ball circumstance [6]. In the case of uncertain wickets, despite the presence of several umpires and a well-known videographer, they had difficulty making timely, precise decisions. Out of the limited research that has been done to detect the no ball, there has not been much using the CNN-based models to solve the problem. In relation to this, the suggested system proposes a newly created dataset since the nonend striker's image data is the key source of information for front no-ball detection. The entire dataset was later pruned while keeping just that portion. The quantity and quality of the data affect both the performance of ML and DL models, thus we employed a variety of pertinent augmentation techniques to increase the data size and certain image enhancement approaches to improve the quality of the images to train a tuned CNN model using keras tuner and a few well-known pretrained models (VGG19, VGG16, ResNet50, InceptionV3, and MobileNet). Here, in this study, VGG16 presented better results in terms of accuracy (0.98), precision, and recall. Thus, the system is designed through data collection, processing, augmentation, modeling, and evaluation.

This study's research challenges are listed as follows:

1. Main challenge was collecting the dataset.
2. Resizing and tuning the image were the next challenge that was undertaken during the study.
3. Modifying and finding the best model parameters.

The key main contributions of this study are given as follows:

1. We initiated the dataset (https://drive.google.com/drive/folders/1_4PFP_zZEifYCnVvhkdBUuzwb03ioQMp?usp=sharing) as there was no available one for detecting no ball by using both manual and automated processes from various online sources, for instance, Google search, highlights, and live matches, and annotated it into two categories such as “legal” and “no ball”.
2. We cropped the images while trimming out unnecessary portions as foot no ball is detected in the striker end.
3. To enlarge the dataset, we used various augmentation techniques such as rotation, width and height shifting, shearing the range, and horizontal flip.
4. We used some image enhancement techniques to make the images sharper and brighter.
5. We implied 5 (five) transfer learning models alongside optimized tuned models trained on the augmented and enhanced images and optimized CNN models are settled by hyperparameter tuning.
6. Finally, we evaluated the model on performance metrics such as accuracy, precision, recall, and F1-score.

The rest of the paper contains Section 2 which is literature review on different research papers, and Section 3 presents an overview of the cricket game.  Section 4 shows the methodology used in the whole process.  Section 5 presents the experimental results and discussion on the generated results, and finally, Section 6 shows the conclusion and the future works.

## 2. Related Works

In recent years, in order to make smart cities [7], researchers have invented a number of technologies. As a result of this idea, smart sports such as smart cricket have become very important. Although we conducted a literature review and observed that there has been minimal deep learning research in cricket no-ball recognition, Rahman et al. [8] developed a unique approach for identifying the kind of delivery from a bowler's finger grip while the bowler is making a delivery. They correctly classify bowlers' grips with 0.9875 accuracy. To prevent umpires from making mistakes owing to human error, Iyer et al. [9] proposed automatic system for deciding run outs and no-ball deliveries.

Here, they tried with different CNN-based model VGG16 and machine learning model SVM for classification; in both the cases, VGG16 outperforms the SVM which shows the power of CNN in extracting the feature from the image data compared to other structures. It detected no ball with an accuracy of 0.8923, and in the case of run, it out achieved an accuracy of 0.8889. Kowsher et al. [10] studied to avoid erroneous interpretations brought on by perspective mistakes, and an automated multidimensional visual system was presented. This work initially has presented a technique for automated no-ball decision-making to distinguish between virtual fault and true decision which aims towards a system which can demolish bad interpretations because of perspective errors by analyzing the team, player performance, and evaluation of playing environments before and after the match to find the insights about the game, players, strategy, and the environments using a graphics system based on computer and by using many dimensions to approximate a ball's movement and contrasting the anticipated path to the main line. CNN models are used thoroughly to counter image-related problems. Namburu et al. [11] investigated the X-ray images with the help of CNN based on several pretrained state-of-art models. An investigation was done by using [12] medical imaging to detect breast cancer using several ML algorithms, and image processing and segmentation techniques are being used by them on the mammogram data of patients. As an extension, Harun-Ur-Rashid et al. [6] employed a CNN-based classification technique using Inception V3 to automatically distinguish and categorize waist high no balls. Their approach achieves an overall average accuracy of 0.88 with a comparatively low cross-entropy value. A thorough examination of the cricket pitch [13] may be useful in forecasting winners and losers while also eliminating the necessity for manual pitch analysis. They have decided to investigate the impact of fractures on the cricket pitch on the ball bowled by bowlers. Minhas et al. [14] investigated an effective shot categorization approach for on-field sport footage based on AlexNet convolutional neural networks (AlexNet CNN) which yielded a 0.9407 accuracy. Khan et al. [15] initiated deep convolutional neural networks based systems to identify and categorize distinct batting strokes from cricket videos. The proposed model can recognize a shot with 0.90 accuracy. Sen et al. [16] initiated a hybrid deep neural network architecture for the classification of 10 distinct cricket batting strokes from offline footage with 0.93 height accuracy. Tong et al. [17] demonstrated the framework (unified) for the types of field sports played with ball for the purpose of shot of semantic in category, which leads to separation of video frames based on three main important factors such as diameter of camera snap, technology used for video creation, and main topic in a scene. They outlined the frameworks, defined semantic shot, and worked with a few instances to provide detection based on the three properties. The results were tested using shot clustering and retrieval, video segmentation (temporal), and semantic video analysis. Li et al. [18] made extension of this work, aiming towards detection of video shots and its implication in detecting events to detect shots on specific game using some predefined rules. They used visual words model to demonstrate the main frame for each individual shot which will go to SVM and PLSA to classify the main frame towards predicting the type of shot, as it is not domain specific and can be integrated with different types of games. Chowdhury et al. [19] used computer vision to detect foot no ball in a cricket match which applied image subtraction method on the pixel value for having the chance to make a judgment. Despite the fact that several tracking methods for improved monitoring of crickets have been published in a number of articles, relatively few studies specifically address cricket no ball tracking. Batra et al. [20] implemented augmented reality for ball tracking and automated no-ball detection where they calculated the distance among bowling crease point, popping crease point, and foot marks of the bowlers using a contour algorithm to label a ball whether no or not.

Therefore, this study aimed towards making an automated system considering only the video content of the bowler's end and popping crease. Hence, it is capable of detecting no ball automatically without intervention of extra devices rather than the one used in cricket matches.

## 3. Cricket Game Overview

Cricket is the world's second popular game, played between two teams. There is unanimity among experts that the history of cricket begins in the late 16th century. It started in the south-east of England, and in the 18th century, it turned into a global sport and expanded internationally between the 19th and 20th centuries. Since the 19th century, international matches have been played, besides official test matches dating back to 1877 [21].  Figure 1 captures a moment of that time. Cricket is internationally conducted by the International Cricket Council (ICC). Cricket rules and laws, such as LBW, stumps, and bat width, were devised and eventually adjusted in 1774 [22]. And as time passes, things begin to shift and evolve, and fresh regulations are added. These regulations and laws were visible on the cricket pitch following the introduction of umpires. And nowadays, it is not simply a game but also an expression of people's emotions. As a result, the impact of a match's outcome is not limited to two countries. However, there are situations when umpires make mistakes that cause a lot of controversy. And classifying a ball as a no ball is a critical choice. There are several examples of this type that have resulted in a significant debate. Once, Lasith Maliinga detected a no ball by a significant margin but the umpire neglected to register it [23]. Another one was done by Ben stokes, where England's fast bowlers conceded 3 consecutive no balls [24] but none of those was marked by the on-field umpires.  Figure 2 depicts the cricket pitch. Out of the 21 types of no balls and their rules, few of those are for front-foot and back-foot no balls. A ball will be considered as no ball if no part of the front foot landed within the area of popping crease, if bowler's back foot touches or landed on the return crease, and 3rd one is if somehow front foot touches the imaginary line of the two middle stumps shown in Figures 3–6, respectively.

## 4. Proposed Methodology

Detecting no-ball with an AI system is all about feeding the model with captured video from left and right side of the ground to make a judgment. In this research paper, we created a dataset and tested the model with video frame after training the model with prepossessed and trimmed data set. A step-by-step workflow diagram in detecting overstepping is given in Figure 7, and the algorithm 1 depicts the pseudo-code.

### 4.1. Dataset

Using the methods described (see Figure 8), we created a dataset of no-ball and legal-ball images:

1. Identifying the research objectives: The first step is to identify the research objectives (see Introduction section).
2. Data sourcing and collecting the images: We collected no-ball and legal-ball images from several publicly available sources such as Google (https://www.google.com), live cricket match (https://www.youtube.com/@TSportsbd), and highlights (https://www.youtube.com/@officialenglandcricket) (see Data Collection section).
3. Annotating and preprocessing the data: The images were labelled after we took to illustrate the location of the no ball and its boundaries according to the rules defined by ICC (https://www.icc-cricket.com) and then we preprocessed the images.
4. Analyzing and evaluating the data: The dataset was split into training, validation, and test sets. After that the training set is used to train the deep learning model; the validation and test sets are used to evaluate the model's performance (see Experimental Results section).

### 4.2. Data Collection

Gathering the data is one of the major parts of the research. And like others, we collected data from Google and by capturing images from the live cricket match and highlights. Images involved in the process were not only from the international but also from domestic practice matches and also from the practice sessions. A sample of raw data is shown in Figure 9 and Table 1 depicts the data distribution among training, validation, and testing set, which is almost balanced.

### 4.3. Data Cropping

The picture region near the nonstrikers is solely significant in the process of identifying no‐ball through over-stepping. The image of the entire playground does not have to be counted while classifying. As a result, cropping all of the images was required immediately after gathering data in order to create this system.  Figure 10 depicts the picture condition after cropping [25].

### 4.4. Data Augmentation

Data augmentation [26] is one of the go to techniques in the image processing types of problem using machine and deep learning. There are many reasons to adopt this in the system. It helps to generate images based on the original images, thus increasing the datasets and enabling models to learn from different perspectives, which further plays a big hand in resolving over-fitting problem [27]. Keeping all that in mind, there are several augmentation techniques implied in this study for making robust models as shown in Table 2.

### 4.5. Data Enhancement

Image enhancement is a key component of strategies for improving image quality, such as emphasizing significant areas and eliminating or weakening distortion or noise in the image [28–30]. Smooth and sharp, noise reduction, deblur pictures, contrast adjustment, brighten an image, and gray‐scale image histogram equalization are some of the prominent ways [31, 32]. Furthermore, the optimum feasible combination of those is essential to keep the system running smoothly.  Figure 11 demonstrates some of those after effects of image enhancement.

### 4.6. Convolutional Neural Network

The convolutional neural network (CNN or convnet) [33] is a significant subgroup of the three artificial neural net-learning models with 100 *∗* 100 dimension. A CNN is a sort of network design for deep-learning algorithms that is mostly used for image classification, identification, localization, and detection tasks that include the handling of pixel input. Convnet is responsible for extracting the feature which defines the image followed by the pooling layer [34], which ends up with a flatten layer [35] to convert higher dimensional data into 1D.  Figure 12 captures the functioning of a CNN.  Table 3 presents the experimental parameters while tuning the hyperparameters.

The number of successfully predicted input data in terms of the total number of samples is referred to as accuracy [36].

(1) $$\begin{array}{c} Accuracy=\frac{TP+TN}{TP+TN+FP+FN}\text{,}\\ Precision=\frac{TP}{TP+FP}\text{,}\\ Recall=\frac{TP}{TP+FN},\\ F1\;score=2\;*\frac{Precision\;*\;Recall}{Precision+Recall}. \end{array}$$

### 4.7. Transfer Learning

Transfer learning is a machine learning approach that entails applying a learning approach produced for one issue as the basis for a model for another [37, 38]. It uses a previously trained model to solve a new problem. Shorter training timeframes, greater artificial neural output (in most circumstances), and the lack of a large quantity of data are indeed the main strengths of transfer learning (TL), VGG19 [39], VGG16 [40], and ResNet50 [41], which is based on the residual network [42]; InceptionV3 [43] and MobileNet [44] are used as pretrained models in this study.  Table 4 depicts the model's parameters.

## 5. Experimental Results and Analysis

This section holds the empirical results obtained by hyperparameter tuned CNN and a few pretrained models after feeding the trained data. Instead of having an almost balanced dataset, models were evaluated based on the classification report [45] (accuracy, precision, recall, and F1-score).  Table 5 demonstrates the performance of the models.

Figure 13 depicts the accuracy of different models in the bar chart. All the 5 (five) pretrained models and the optimized CNN perform quite well in learning the features of the images and classifying them with the highest classification rate of 0.98 is achieved jointly by both VGG19 and VGG16.

ResNet 50 performed relatively low as compared to others. And Table 6 depicts the empirical macro and weighted average. All the models trained for 50 epochs using the available GPU of Google colab and kept track of model training progress. The accuracy of each model increases as epochs go. The over-fitting is a common issue, and most of the time, the training occurs when there is a good amount of gap between validation and training accuracy.  Figure 14 demonstrates that VGG19 was slightly over-fitted [46] as epochs go. And VGG16 seems smoother in terms of training and validation accuracy.

Figure 15 shows the confusion matrix [47] of all the models, which is also a powerful tool for evaluating models based on their reactions to positive and negative categories. The value in the top right-hand corner box represents the false positive, whereas the value in the bottom left corner box denotes the false negative and the FN value is quite low, ranging between 0 and 2, indicating that the models identify the no ball correctly but are a little perplexed in determining the legal ball. Finally, it would not be incorrect to state that the system works well and reliably enough to discern between legitimate and illegal deliveries.

Finally, after reviewing all the pertinent works, although currently there is not enough research in this area. Here, it summarizes the comparison among related works.

1. Chowdhury et al. [19] applied the image subtraction method to the pixel value for having the chance to make a judgment by further testing the system for 6 input frames using computer vision, where our proposed system is tested on 262 test images.
2. Batra et al. [20] introduced a no-ball detection system through the distance among bowling crease points, popping crease point, and foot marks of the bowlers using the contour algorithm. On the contrary, deep learning models are implied as the classifier in our proposed method and have achieved reliable satisfactory results.
3. Harun-Ur-Rashid [6] built a framework using CNN and Inception V3 models including image processing techniques to segregate waist-high no ball and legal deliveries and achieved 0.92 accuracy compared to which this framework started with data collection, augmentation, enhancement, modeling, and evaluation with test data and counted 0.98 accuracy.

## 6. Conclusions and Future Works

In this study, a deep learning-based approach was proposed to detect no balls in cricket. The study began with a thorough background study to gather domain information, followed by the creation of a dataset containing two classes: legal and no ball which was then segregated into training, validation, and test sets. Various image augmentation techniques were applied to increase the dataset's size and create a robust model. Additionally, image enhancement techniques were used to make the images brighter and clearer. The performance of a fine-tuned CNN model and a modified state-of-the-art pretrained model were compared, and the selected VGG16 model achieved a 0.98 accuracy rate.

The findings of this study could potentially give cricket organizations and policymakers information on the effects of technology on the fan experience. Decisionmakers should consider the potential effects on fan engagement, motivation, and loyalty before deciding whether to deploy no-ball detection systems or other similar technologies. Moreover, the study could aid in formulating plans to mitigate any negative effects on the fan experience and keep fans engaged despite technological progress.

Despite the proposed system's success, it has some drawbacks, including real-time identification from video frames, training models on large amounts of data, and the use of sophisticated picture enhancing methods. These limitations suggest potential future applications to increase the dataset's size and incorporate enhancement techniques such as histogram equalization, noise removal using a Wiener filter, linear contrast adjustment, median filtering, and unsharp mask filtering. Integrating this system with the video camera of cricket grounds and incorporating a voice assistant system for taking immediate actions as soon as a no ball is detected could also be explored. Additionally, amalgamating evidential reasoning [48, 49], adopting belief rule-based systems [50–52] with deep learning models, and employing explainable artificial intelligence (XAI) [53] technologies could potentially yield better outcomes.

## Figures and Tables

**Figure 1:** Cricket history.

**Figure 2:** Cricket pitch.

**Figure 3:** Crossing popping crease.

**Figure 4:** Touching return crease.

**Figure 5:** Landing on imaginary line.

**Figure 6:** No‐ball.

**Figure 7:** Outline of the performed experiment.

**Figure 8:** Steps involved in creating an image dataset.

**Figure 9:** Front foot no‐ball.

**Figure 10:** Cropped image.

**Figure 11:** Data enhancement.

**Figure 12:** Convolutional neural network.

**Figure 13:** Accuracy comparison among the models.

**Figure 14:** Accuracy graph while training. (a) Optimized-CNN. (b) VGG19. (c) VGG16. (d) ResNet 50. (e) Inception V3. (f) MobileNet.

**Figure 15:** Confusion matrix. (a) Optimized-CNN. (b) VGG19. (c) VGG16. (d) ResNet 50. (e) Inception V3. (f) Mobile net.

**Algorithm 1:** Algorithm for detecting no‐ball.

**Table 1:** Dataset distribution.

Datasets	Number of images		
	No balls	Legal balls	Total images
Train data	1463	1200	2663
Validation data	190	180	370
Test data	133	129	262

**Table 2:** Data augmentation.

Augmentation techniques	Parameters
Centering	featurewise_center = true
Normalization	featurewise_std_normalization = true
Rotation	rotation_range = 20
Width shift	width_shift_range = 0.1
Height shift	height_shift_range = 0.1
Shear	shear_range = 0.3
Flip	horizontal_flip = true

**Table 3:** Parameter configuration.

Parameter configuration	Values
Input image size	100 *∗* 100
Pooling layer	Max-polling
Dropout layer	Dropout
Fully connected layer	Flatten
Fully connected layer	Dense
Filter numbers	16, 32, 64
Filter size	3 *∗* 3
Optimizer	Adam
Learning rate	0.001
Loss function	Categorical crossentropy

**Table 4:** Parameters of TL models.

Models	Total parameters	Trainable parameters	Nontrainable parameters
VGG19	20,033,602	9,218	20,024,384
VGG16	14,723,906	9,218	14,714,688
ResNet50	23,653,250	65,538	23,587,712
Inceptionv3	21,806,882	4,098	21,802,784
MobileNet	3,247,298	18,434	3,228,864

**Table 5:** Performance of all the pretrained and tuned CNN.

Models	Accuracy	Precision	Recall	F1-score
Optimised CNN	0.97	0.96	0.99	0.97
VGG19	0.98	0.96	0.99	0.98
VGG16	0.98	0.96	1.0	0.98
ResNet50	0.84	0.77	0.98	0.86
Inceptionv3	0.97	0.94	0.99	0.97
MobileNet	0.97	0.95	0.98	0.97

**Table 6:** Macro and weighted average of the models.

Models	Macro avg		Weighted avg				Accuracy
	Precision	Recall	F1-score	Precision	Recall	F1-score	
Optimised CNN	0.97	0.97	0.97	0.97	0.97	0.97	0.97
VGG19	0.98	0.98	0.98	0.98	0.98	0.98	0.98
VGG16	0.98	0.98	0.98	0.98	0.98	0.98	0.98
ResNet50	0.87	0.84	0.84	0.87	0.84	0.84	0.84
InceptionV3	0.97	0.97	0.97	0.97	0.97	0.97	0.97
MobileNet	0.97	0.97	0.97	0.97	0.97	0.97	0.97

## Data Availability

The data used to support the findings of this study are available upon reasonable request to the corresponding author.
